This article has been retracted.

# The silencing of long non-coding RNA ANRIL suppresses invasion, and promotes apoptosis of retinoblastoma cells through the ATM-E2F1 signaling pathway

**DOI:** 10.1042/BSR20180558

**Published:** 2018-12-11

**Authors:** Yang Yang, Xiao-Wei Peng

**Affiliations:** Department of Pediatric Ophthalmology, The Second Affiliated Hospital of Nanchang University, Nanchang 330006, P.R. China

**Keywords:** ATM-E2F1 signaling pathway, Cell apoptosis, Cell proliferation, Long-non coding RNA ANRIL, Negative feedback regulation, Retinoblastoma

## Abstract

As one of the most common primary intraocular carcinomas, retinoblastoma generally stems from the inactivation of the retinoblastoma *RB1* gene in retinal cells. Antisense non-coding RNA in the INK4 locus (ANRIL), a long non-coding RNA (lncRNA), has been reported to affect tumorigenesis and progression of various cancers, including gastric cancer and non-small cell lung cancer. However, limited investigations emphasized the role of ANRIL in human retinoblastoma. Hence, the current study was intended to investigate the effects of ANRIL on the proliferation, apoptosis, and invasion of retinoblastoma HXO-RB_44_ and Y79 cells. The lentivirus-based packaging system was designed to aid the up-regulation of ANRIL and ATM expressions or employed for the down-regulation of ANRIL in human retinoblastoma cells. Afterward, ANRIL expression, mRNA and protein expression of ATM and E2F1, and protein expression of INK4b, INK4a, alternate reading frame (ARF), p53 and retinoblastoma protein (pRB) were determined in order to elucidate the regulation effect associated with ANRIL on the ATM-E2F1 signaling pathway. In addition, cell viability, apoptosis, and invasion were detected accordingly. The results indicated that the down-regulation of ANRIL or up-regulation of ATM led to an increase in the expressions of ATM, E2F1, INK4b, INK4a, ARF, p53, and pRB. The silencing of ANRIL or up-regulation of ATM exerted an inhibitory effect on the proliferation and invasion while improving the apoptosis of HXO-RB_44_ and Y79 cells. In conclusion, the key observations of our study demonstrated that ANRIL depletion could act to suppress retinoblastoma progression by activating the ATM-E2F1 signaling pathway. These results provide a potentially promising basis for the targetted intervention treatment of human retinoblastoma.

## Introduction

Retinoblastoma is an aggressive form of an intraocular cancer usually occurring during childhood that is initiated by the mutation of the *RB1* gene. Timely diagnoses along with early treatment may boast excellent outcome, however, retinoblastoma may also be a life-threatening condition if left without a swift and adequate treatment [1,2]. Although the etiology of retinoblastoma is relatively well-understood, the mortality rate of the condition sits at an alarming 70% in lower and middle-income countries (MICs); while the incidence rate of retinoblastoma has been found to be higher amongst Asian and African regions, and children were reported to have a greater susceptibility to it with a mortality rate of approximately 40–70% [3]. An investigation into retinoblastoma survival in less-developed countries, suggested there to be an estimated survival rate of 40% in lower income countries with survival rates approximately 77% and 79% in lower MICs and upper MICs, respectively [4]. The treatment for retinoblastoma generally includes ophthalmectomy, chemotherapy, laser photocoagulation, plaque radiotherapy, thermotherapy, and external radiotherapy, while over the past 2 years, intra-arterial chemotherapy, a novel treatment for retinoblastoma, has been evaluated and appeared to have superior curative effects [5].

Long non-coding RNAs (lncRNAs), range in length from 200 to 100000 nts, do not possess the ability of being translated into proteins, represent regulatory RNA that play significant roles in the process of cell differentiation and development [6,7]. Studies have shown that lncRNAs are associated with the pathogenesis of various conditions including cancer, while the dysregulation of lncRNAs has also been reported to exist in various types of human cancers, including prostate cancer, gastric cancer, and recently, retinoblastoma [8–11]. Antisense non-coding RNA in the INK4 locus (ANRIL), which belongs to the lncRNA family, is widespread in many kinds of human tumors, and has also been considered to be a dangerous factor in breast cancer as well as several other cancers by accumulating studies. ANRIL knockdown was reported to have an inhibitory effect on proliferation either *in vivo* or *in vitro* [12,13]. Other studies have also demonstrated that that ANRIL expression, which was induced through ATM-E2F1 signaling pathway, increased notably in gastric cancer tissues and non-small cell lung cancer tissues, with reports highlighting its ability to promote proliferation while inhibiting the apoptosis of cancer cells [10,14]. The ATM kinase is a key sensor in the DNA damage response pathway that responds particularly to dsDNA breaks and the most severe genomic damage, and ATM-mediated phosphorylation of downstream target proteins triggers cascade signals resulting in the activation of DNA repair and cell cycle checkpoints [7]. The ANRIL expression is regulated by ATM-E2F1 signaling pathway, and its activation was induced by E2F1 transcriptionally, such activation was induced by ATM and fulfilled by the mediation of E2F1 activation, an important tumor suppressor [7]. As a result, it is of great significance to further investigate the role of ANRIL in the biological processes of retinoblastoma cells. Thus, the current study was conducted in order to evaluate the effects associated with the specific lncRNA and ANRIL on regulating the biological processes involved in human retinoblastoma cells, including proliferation, apoptosis, and invasion, while further exploring the potential regulatory role and involvement of the ATM-E2F1 signaling pathway.

## Materials and methods

### Cell culture

Human retinoblastoma HXO-RB_44_ and Y79 cells were purchased from the Institute of Biochemistry and Cell Biology, Shanghai Institutes for Biological Sciences, Chinese Academy of Sciences (Shanghai, China). Cells preserved in liquid nitrogen in a sealed tube were taken out and rapidly thawed in a water bath at 37°C. Following sterilization using 75% ethanol, the cell sap in the sealed tube was transferred to a centrifuge tube containing Eagle’s minimum essential medium (EMEM) using a clean bench (Thermo Fisher, CA, U.S.A.), after which it was centrifuged at 290×***g*** at 4°C for 3 min. The supernatant was then carefully removed with the cells then re-suspended and transferred to a culture flask (Corning Inc., NY, U.S.A.) containing EMEM supplemented with 10% FBS and 1% double antibody (Gibco, NY, U.S.A.). The cells were subsequently incubated in an incubator containing 5% CO_2_ at 37°C. When the cells had reached approximately 70–80% confluence, they were treated with trypsin and passed into six-well plates with the density adjusted to 1 × 10^5^ cells/well.

### Construction of vectors

Based on the full length of 1258 bp cDNA sequence of ANRIL obtained from the NCBI (GI: 641451086), the specific primers of target genes were designed and restriction enzyme Xba I and BamH I recognition sites were introduced. Reverse transcription quantitative PCR (RT-qPCR) methods were performed for amplification purposes with the recovered purified PCR products subsequently inserted into the pMD18-T vector (TaKaRa Biotechnology Co. Ltd., Liaoning, China) and transformed into *Escherichia coli* (*E. coli*) DH5α competent cells. After the positive clones were obtained by means of blue-white screening, the plasmids were extracted and confirmed by means of restricted digestion. Lentiviral vector pCD513B (System Biosciences Inc., CA, U.S.A.) carrying GFP as well as the puromycin resistance gene were used for ANRIL overexpression. The pCD513B vector was then linearized after the digestion of the restriction enzymes Xba I and BamH I, and the target gene fragments and the linearized vector ligated with T4 DNA ligase, after which the ligation mixture was transformed into *E. coli* DH5α competent cells. After the positive cloned cells were selected by virtue of the ampicillin resistance, plasmid extraction and identification was performed by means of Xba I and BamH I enzymes digestion. The method for the vector construction of overexpressed ANRIL was also applied to the vector construction of ATM. ANRIL-shRNA was transfected into cells in order to silence ANRIL using a Lipofectamine™ 2000, with ANRIL NC regarded as the control.

### Cell transfection and grouping

Cells at the exponential phase were seeded in six-well plates (approximately 1–3 × 10^5^ cells/well) and cultured with CO_2_ overnight until the cells were confirmed to have reached 50–80% confluence. Next, the cells were assigned into six groups, namely control group (without any transfection), negative control (NC) group (transfected with empty vectors), overexpressed ANRIL group, sh-ANRIL group (transfected with ANRIL-shRNA), overexpressed ATM group, and overexpressed ATM + overexpressed ANRIL group. The following solutions were prepared in a simultaneous manner: (A) 100 µl serum-free medium added with 1–2 µg high quality vector DNA; (B) 100 µl serum-free medium added with 1–2 µl Lipofectamine 2000 (Invitrogen Inc., CA, U.S.A.). Solutions A and B were mixed and placed at room temperature for 15–45 min in order to facilitate the formation of DNA–liposome complex. A total of 2 ml serum-free medium was used to wash the cells and 0.8 ml serum-free medium was added into the DNA–liposome complex. The mixture was then gently shaken in a thorough manner and then slowly added dropwise into the six-well plates, followed by incubation in an incubator containing 5% CO_2_ for over 6 h. Each six-well plate was then added with 1 ml medium with double concentration of serum and the culture containing serum then refreshed following a 24-h period of transfection. The total RNA and protein were extracted over a 72-h period post transfection.

### RT-qPCR

The total RNA was extracted using TRIzol (Takara, Kyoto, Japan) from the cells at the 72 h point after transfection. The optical density (OD) value and OD260/280 ratio were measured using a micro-spectrophotometer (NanoDrop Technologies, DE, U.S.A.) after which cDNA was synthesized using a reverse transcription kit (Takara, Kyoto, Japan). The primers for ANRIL, ATM, and E2F1 were synthesized by Shanghai Sangon Biological Engineering Technology and Services Co., Ltd., (Shanghai, China), as illustrated in Table 1. The SYBR Green Real-time Fluorescence Quantitative PCR Kit was applied in order to determine the total volume of reaction system which was confirmed to be 20 μl. Glyceraldehyde-3-phosphate-dehydrogenase (GAPDH) was considered to be the internal reference. The reaction system and conditions are illustrated in Tables 2 and 3. The quantitative results were calculated based on the method 2^−ΔΔ*C*^_t_ which demonstrated the relative gene expression ratio of the experimental group to the control group. The formula of 2^−ΔΔ*C*^_t_ method was as follows: ΔΔ*C*_T_ = Δ*C*_t__experimental group_ − Δ*C*_t__control group_; Δ*C*_t_ = *C*_t__target gene_ − *C*_internal reference_.

**Table 1:** Primer sequences of ANRIL, ATM, E2F1, and GAPDH for RT-qPCR

Gene	Sequence (5′–3′)
*ANRIL*	F: TTGTGAAGCCCAAGTACTGC
	R: TTCACTGTGGAGACGTTGGT
*ATM*	F: TGGATCCAGCTATTTGGTTTGA
	R: CCAAGTATGTAACCAACAATAGAAGAAGTAG
*E2F1*	F: ACCAGGGTTTCCAGAGATGC
	R: CACCACACAGACTCCTTCCC
*GAPDH*	F: AGAAGGCTGGGGCTCATTTG
	R: AGGGGCCATCCACAGTCTTC

Abbreviations: F, forward; R, reverse.

**Table 2:** Reaction system of RT-qPCR

Component	Volume
Forward primer	1.0 µl
Reverse primer	1.0 µl
SYBR® Premix Ex Taq™	10 µl
(10×) cDNA	6 µl
DEPC water	2 µl

Abbreviation: DEPC, diethylpyrocarbonate.

**Table 3:** Reaction conditions of RT-qPCR

Cycle	Procedure
Hold @ 95°C, 2 min 0 s	
	Step 1 @ 95°C, hold 10 s
Cycling (40 repeats)	Step 2 @ 60°C, hold 30 s
	Step 3 @ 70°C, hold 30 s, acquiring to Cycling
Melt (70–95°C)	

### Western blot analysis

After transfection for 72 h, the protein levels of ATM, E2F1, INK4b, INK4a, alternate reading frame (ARF), p53 and retinoblastoma protein (pRB) were detected by Western blot analysis, with GAPDH employed as the internal reference. The total proteins were extracted with the protein concentration then determined accordingly. Spacer gel and separating gel were prepared and loading quantity of sample was set. The spacer gel ran at 60 V, which was then turned up to 100 V, followed by a wet-transfer process at 100 V for 70 min with the proteins transferred to the membrane. Membrane blockade was then conducted using a mixture containing 10% skim milk powder and TBS for 2 h after which the membrane was incubated overnight at 4°C with the addition of the following diluted primary antibodies: Anti-ATM (p-S1981), Anti-E2F1 (KH95), Anti-p15 INK4b, Anti-CDKN2A/P16-INK4a [EPR1743], Anti-CDKN2A/P14- ARF [ARF4C6/4], Anti-p53 [DO-1], Anti-PRB1/2 [EPR7927], and Anti-GAPDH (Abcam, Cambridge, U.K.). After rewarming for 2 h at room temperature, the membrane was washed five times with PBS containing 0.1% Tween-20 (PBST) every 8 min. Afterward, the membranes were incubated with horseradish peroxidase-labeled anti-rabbit second antibody (CalBiochem, Bad Soden, Germany) at room temperature for 2 h. The membranes were then further washed five times with PBST at 8-min intervals. Finally, an electrochemiluminescence assay was performed.

### Cell counting kit-8 assay

The transfected cells were seeded in a 96-well plate at a density of 4 × 10^3^ cells/100 µl, with each well supplemented with 20 µl Cell counting kit-8 (CCK-8) solutions. After incubation for 4 h, the supernatant was removed, followed by gentle shaking with the addition of 150 µl DMSO in each well for 10 min. An OD value at 499 nm was subsequently determined using an enzyme-labeling measuring instrument (Bio-Tek, VT, U.S.A.), and then the cell proliferation curves were constructed with the x-axis representing time and y-axis representing OD value.

### Flow cytometry

Annexin V/propidium iodide (PI) double staining was performed in order to determine cell apoptosis, while HXO-RB_44_ cells at the logarithmic phase of growth were adopted. The adopted HXO-RB_44_ cells were then suspended following detachment with 0.25% trypsin and were seeded in culture plate with a density of 1 × 10^5^ cells/ml, after which they were washed three times with pre-cooled PBS at 4°C and treated with trypsin. Following 5 min of centrifugation at 290×***g***, the supernatant was removed and the cells were re-suspended with PBS. The concentration of the transfected cells was adjusted to 1 × 10^6^ cells/ml. A total of 100 µl cell suspension was centrifuged at 290×***g*** for 5 min, after which the supernatant was discarded and 500 µl 1× binding buffer, 5 µl FITC-labeled annexin V (annexinV-FITC), and 10 µl PI were added in a successive manner, followed by gentle shaking. The mixture was incubated at room temperature for 5–10 min under conditions void of light with a flow cytometer (BDLSR II, BD Biosciences, Franklin Lakes, NJ, U.S.A.) subsequently employed cell apoptosis analysis purposes. A total of 100 µl of cell suspension was centrifuged at 290×***g*** for 5 min after which the supernatant was discarded, washed twice with pre-cooled 200 µl PBS, and treated with 20 µl RNase at 37°C for 30 min. Next, the cells were incubated with 400 µl PI (C0080, Beijing Solarbio Science & Technology Co., Ltd. Beijing, China) on ice under conditions void of light for 15 min. Finally, cell cycle was detected using flow cytometer (BDLSR II, BD Biosciences, Franklin Lakes, NJ, U.S.A.) at an excitation wavelength of 488 mm.

### Transwell assay

A total of 20–30 µl of Matrigel was added into each well of the filter membrane of the chamber at 37°C overnight with fibronectin added in an even manner to the other side of the membrane. Next, 1 × 10 ^5^ cells were added in the Transwell chamber. After a 24-h period of incubation, the cells on the upper layer of membrane were removed and the membrane was obtained and subsequently fixed with formaldehyde and placed at room temperature for 30 min. Next, the cells were stained with Hematoxylin for 3–5 min, dehydrated with ethanol (5 min each time), and cleared with formaldehyde. A portion of the lower layer of membrane was subsequently selected and placed on a slide for further observation, with the average of four representative views selected followed by cell number counting under a microscope.

### Statistical analysis

Statistical analysis was performed using SPSS 18.0 software (IBM Corp. Armonk, NY, U.S.A.). Categorical data were measured by chi-square test and the measurement data were expressed as mean ± S.D. One-way ANOVA was employed for the comparisons of multiple groups. A *P*-value <0.05 was considered to be indicative of statistical significance.

## Results

### Successful construction and transfection of T-ANRIL and pCD513B-ANRIL vectors

Initially, T-ANRIL, an ANRIL cDNA clone, was constructed. After digestion by restriction enzymes Xba I and BamH I, the bands of 1700 and 1400 bp were observed accordingly. The length of pMD18-T was determined to be approximately 2700 bp with the full length of the ANRIL cDNA approximately 1400 bp. T-ANRIL was successfully constructed, as illustrated Figure 1A. The two bands of approximately 8000 and 1400 bp of pCD513B-ANRIL, a vector for ANRIL overexpression, were observed following the digestion of restriction enzymes Xba I and BamH I. The length of linearized vector pCD513B was approximately 8100 bp, while the full length of ANRIL cDNA was approximately 1400 bp. As depicted in Figure 1B, pCD513B-ANRIL was successfully constructed. As GFP was carried by the pCD513B-ANRIL, green fluorescence in HXO-RB_44_ could be observed under a fluorescence microscope in the event that the cells were transfected. The transfection of HXO-RB_44_ is illustrated in Figure 1C. No fluorescence appeared in the cells without transfection under a fluorescent microscope (Figure 1D). Thus, T-ANRIL and pCD513B-ANRIL vectors were deemed to be successfully constructed.

**Figure 1:** T-ANRIL and pCD513B-ANRIL vectors were successfully constructed while the HXO-RB44 cells were successfully transfected and subsequently observed under a fluorescence microscope (**A**) 250 bp DNA marker; (**B**) 1000 bp DNA marker; (**C**) green fluorescence in post-transfected cells under fluorescence microscope (40×); (**D**) non-transfected cells under fluorescence microscope (40×).

### ANRIL negatively regulates the ATM-E2F1 signaling pathway

RT-qPCR and Western blot analysis were employed for observation of the regulatory roles of ANRIL in the ATM-E2F1 signaling pathway. ANRIL expression and mRNA and protein levels of ATM and E2F1 were detected amongst the five groups with GAPDH considered as the internal reference, the results of which are depicted in Figure 2. Compared with the control and NC groups, a remarkable increase in the ANRIL expression and a reduction in ATM and E2F1 mRNA and protein levels amongst the cells in the overexpressed ANRIL group were observed (both *P*<0.01). The sh-ANRIL group exhibited decreased in ANRIL expression (*P*<0.05) along with decreased mRNA and protein expression of ATM and E2F1 (both *P*<0.05). The mRNA and protein levels of ATM and E2F1 were significantly higher in cells of the overexpressed ATM group (all *P*<0.01), while there were no notable variations observed regarding the expression of ANRIL (*P*>0.05). In the overexpressed ATM + overexpressed ANRIL group, the ANRIL expression was markedly increased when compared with the control and NC group (*P*<0.05), while the *ATM* and *E2F1* mRNA and protein levels were similar to those in the control group (*P*>0.05). These findings indicated that ANRIL could down-regulate the ATM-E2F1 signaling pathway.

**Figure 2:** The ATM-E2F1 signaling pathway was down-regulated by ANRIL based on the RT-qPCR and Western blot analysis (**A**) Relative mRNA levels of ANRIL, ATM, and E2F1 in HXO-RB_44_ cell line in each group; (**B**) protein bands of ATM and E2F1 and protein expression of ATM and E2F1 in HXO-RB_44_ cell line in each group; (**C**) the mRNA expression of ANRIL, ATM, and E2F1 in Y79 cell line in each group; (**D**) protein bands of ATM and E2F1 and protein expression of ATM and E2F1 in Y79 cell line in each group; *, *P*<0.05 compared with the control and NC groups; **, *P*<0.01 compared with the control and NC groups. Measurement data were expressed as mean ± S.D., comparisons amongst multiple groups were performed by one-way ANOVA, and the experiment was repeated three times.

### ANRIL silencing inhibits proliferation of retinoblastoma cells

CCK-8 assay was conducted in order to determine the effect of ANRIL on the proliferation of HXO-RB_44_ and Y79 cells, while subsequently comparing the viability of transfected cells amongst 12 groups. As shown in Figure 3, on the sixth day, the cell viability increased in the overexpressed ANRIL group, while it decreased in the sh-ANRIL group and the overexpressed ATM group (all *P*<0.05) when compared with the control and NC groups; no significant difference was detected in the overexpressed ATM + overexpressed ANRIL group (*P*>0.05). These results demonstrated that ANRIL silencing could act to suppress the cell proliferation of HXO-RB_44_ and Y79 by activating the ATM-E2F1 signaling pathway.

**Figure 3:** ANRIL silencing inhibited the viability of HXO-RB_44_ cells (left) and Y79 cells (right) *, *P*<0.05 compared with the control and NC groups; **, *P*<0.01 compared with the control and NC groups. Measurement data were expressed as mean ± S.D., comparisons amongst multiple groups were performed by one-way ANOVA, and the experiment was repeated three times.

### ANRIL silencing improves apoptosis of retinoblastoma cells

Annexin V/PI double staining method and flow cytometry were performed in order to evaluate the effects of ANRIL on the regulation of HXO-RB_44_ and Y79 cell apoptosis (Figure 4). In comparison with the apoptotic index in the control and NC groups, overexpressed ANRIL group exhibited a remarkable reduction (*P*<0.01), and the sh-ANRIL group as well as the overexpressed ATM group displayed a significant increase (all *P*<0.05). The apoptotic index of the overexpressed ATM + overexpressed ANRIL group was observed to be strikingly similar to that of the control and NC groups (both *P*>0.05). The aforementioned findings suggested that ANRIL silencing promoted the apoptosis of HXO-RB_44_ and Y79 cells by activating the ATM-E2F1 signaling pathway.

**Figure 4:** Down-regulated ANRIL promoted the apoptotic index of HXO-RB_44_ cells and Y79 cells by Annexin V/PI double staining method and flow cytometry (**A**) The cell apoptosis of HXO-RB_44_ cells in each group examined by flow cytometry; (**B**) the cell apoptotic index of HXO-RB_44_ cells in each group; (**C**) the cell apoptosis of Y79 cells in each group examined by flow cytometry; (**D**) the cell apoptotic index of Y-79 cells in each group; *, *P*<0.05 compared with the control and NC groups; **, *P*<0.01 compared with the control and NC groups. Measurement data were expressed as mean ± S.D., comparisons amongst multiple groups were performed by one-way ANOVA, and the experiment was repeated three times.

### Down-regulated ANRIL arrests retinoblastoma cell cycle progression

Flow cytometry was applied in order to examine cell cycle and to determine the DNA content of the single cell in samples, followed by the detection of the cell ratio in G_0_/G_1_, S, and G_2_/M phases. The results (Figure 5) revealed that compared with the control and NC groups, the overexpressed ANRIL group exhibited a lower cell ratio at the G_0_/G_1_ phase but a higher cell ratio at the S phase (all *P*<0.05). The sh-ANRIL group and the overexpressed ATM group displayed a higher cell ratio at the G_0_/G_1_ phase but a lower cell ratio at the S phase in contrast with the control and NC groups (all *P*<0.05). The cell ratio in each phase of the overexpressed ATM + overexpressed ANRIL group was observed to be similar to that of the control and NC group (all *P*>0.05). Thus, based on our results we concluded that ANRIL depletion led to the inhibition of the HXO-RB_44_ and Y79 cell cycle progression by activating the ATM-E2F1 signaling pathway.

**Figure 5:** Down-regulated ANRIL arrested cell cycle progression of HXO-RB_44_ cells and Y79 cells (**A**) Cell cycle of HXO-RB_44_ cells in each group examined by flow cytometry; (**B**) cell ratio of HXO-RB_44_ cells in each phase; (**C**) cell cycle of Y79 cells in each group examined by flow cytometry; (**D**) cell ratio of Y79 cells in each phase; *, *P*<0.05 compared with the control and NC groups; **, *P*<0.01 compared with the control and NC groups. Measurement data were expressed as mean ± S.D., comparisons amongst multiple groups were performed by one-way ANOVA, and the experiment was repeated three times.

### The down-regulation of ANRIL inhibits the invasion of retinoblastoma cells

During the following experiments, the roles of ANRIL in the invasion of retinoblastoma HXO-RB44 and Y79 cells was detected using a Transwell assay. As depicted in Figure 6, compared with the control group and the NC group, invasion of HXO-RB44 and Y79 cells in the overexpressed ANRIL group was significantly higher (*P*<0.01) while it was notably weakened in the sh-ANRIL group (*P*<0.05) and the overexpressed ATM group (*P*<0.01). In the overexpressed ATM + overexpressed ANRIL group, there was no significant difference in regard to the cell invasion ability between the control and NC groups (*P*>0.05). The results indicated that invasion ability of HXO-RB44 and Y79 cells was inhibited by ANRIL silencing.

**Figure 6:** Down-regulated ANRIL suppressed the invasion ability of HXO-RB_44_ cells and Y79 cells as illustrated by Transwell assay (**A**) HXO-RB_44_ cells stained by Crystal Violet in Transwell chamber of each group (×200); (**B**) the cell invasion of HXO-RB_44_ cells in each group; (**C**) Y79 cells stained by Crystal Violet in Transwell chamber of each group (×200); (**D**) the cell invasion of Y79 cells in each group; *, *P*<0.05 compared with the control and NC groups; **, *P*<0.01 compared with the control and NC groups. Measurement data were expressed as mean ± S.D., comparisons amongst multiple groups were performed by one-way ANOVA, and the experiment was repeated three times.

### Protein levels of INK4b, INK4a, ARF, p53, and pRB are increased by ANRIL silencing

At last, Western blot analysis was performed in order to determine the levels of INK4b, INK4a, ARF, p53, and pRB amongst the six groups using GAPDH as an internal reference. As illustrated in Figure 7, the results obtained demonstrated that compared with the control and NC groups, the overexpression of ANRIL as well as the protein levels of INK4b, INK4a, ARF, p53, and pRB decreased in the overexpressed ANRIL group (all *P*<0.05), while that of INK4b, INK4a, ARF, p53, and pRB increased in the sh-ANRIL group and the overexpressed ATM group (all *P*<0.05). However, regarding the protein levels in the overexpressed ATM + overexpressed ANRIL group, there was no significant difference detected in comparison with the control and NC groups (*P*>0.05). The aforementioned results provided evidence suggesting that down-regulation of ANRIL or activation of ATM-E2F1 signaling pathway resulted in increased levels of INK4b, INK4a, ARF, p53, and pRB.

**Figure 7:** Down-regulated ANRIL increased protein levels of INK4b, INK4a, ARF, p53, and pRB detected by Western blot analysis (**A**) Gray value of INK4b, INK4a, ARF, p53, and pRB of HXO-RB_44_ cells in each group; (**B**) protein expression of INK4b, INK4a, ARF, p53, and pRB of HXO-RB_44_ cells in each group; (**C**) gray value of INK4b, INK4a, ARF, p53, and pRB of Y79 cells in each group; (**D**) protein expression of INK4b, INK4a, ARF, p53, and pRB of Y79 cells in each group; *, *P*<0.05 compared with the control and NC groups; **, *P*<0.01 compared with the control and NC groups. Measurement data were expressed as mean ± S.D., comparisons amongst multiple groups were performed by one-way ANOVA, and the experiment was repeated three times.

## Discussion

The vectors for the overexpression of ANRIL and ATM were successfully constructed followed by the negative feedback regulation of the ATM-E2F1 signaling pathway by ANRIL. Through the application of RT-qPCR and Western blot analysis methods, the effects of ANRIL on the regulation of the proliferation, apoptosis, and invasion of retinoblastoma HXO-RB_44_ cells were examined through the ATM-E2F1 signaling pathway. The obtained results demonstrated that ANRIL could influence the biological processes of proliferation, apoptosis, and invasion of the HXO-RB_44_ cells owing to its ability to negatively regulate the ATM-E2F1 signaling pathway. Regardless of the wide spanning knowledge of the etiology of retinoblastoma, the mortality rate remains high at approximately 40% [3]. Previous studies have implicated lncRNAs such as lncRNA BANCR and lncRNA HOTAIR in cases of retinoblastoma with poor prognoses due to their ability to facilitate cell proliferation and invasion [15,16].

Our findings demonstrated that the silencing of ANRIL resulted in the inhibition of retinoblastoma HXO-RB_44_ and Y79 cell proliferation, cell invasion ability, and promotion of apoptosis. A previously conducted study regarding the gastric cancer suggested that the up-regulation of ANRIL had the capability to facilitate the proliferation of cells and suppress cell apoptosis [14]. Similarly, ANRIL was found to strengthen cancer cell invasion and inhibit cell apoptosis, while the up-regulation of ANRIL could promote the hypoxic osteosarcoma cell invasion and inhibit cell apoptosis [17]. A key observation of our study revealed that, ATM overexpression could stimulate an increase in E2F1 expression. In cases where DNA damage is observed, activated ATM and ATR phosphorylation activated the transcription factor E2F1 and thus maintained the stability of the genome [18]. Reports have indicated that the up-regulation of E2F1 induces the expression of ANRIL, leading to the formation of a positive feedback loop, resulting in the continuation of gastric cancer cell proliferation [10]. ANRIL has been shown to be activated through the mutation of kinase-E2F1 transcription factor signaling pathway by the ataxia telangiectasia [19]. The silencing of ANRIL could potentially inhibit cell proliferation, migration, and invasion in hepatocellular carcinoma [20]. E2F1, an effector of the retinoblastoma tumor suppressor pathway was shown to induce suppression of apoptosis with a activation of DNA repair [21]. Moreover, overexpressed ANRIL down-regulated ATM and E2F1, suggesting that ANRIL negatively regulates the ATM-E2F1 signaling pathway. Based on the aforementioned findings, we subsequently concluded that silencing ANRIL suppresses cell proliferation, cell invasion ability, while acting to promote the apoptosis of retinoblastoma cells with a possible involvement of the ATM-E2F1 signaling pathway.

We also found that the underexpressed ANRIL or activated ATM-E2F1 signaling pathway could result in increased expressions of INK4b, INK4a, p53, and pRB. Two major tumor suppressors, the transcription factor p53 and pRB take control of cellular reaction as potential carcinogenic stimuli like the repeated division of cells, damage of DNA as well as improper mitogenic signals and their reactivation significantly takes part in tumor therapy [22,23]. With regard to the expressions of protein-coding genes, ANRIL, the antisense non-coding RNA of the INK4b-ARF-INK4a locus plays a central role [9]. ANRIL was transcribed from the INK4b-ARF-INK4a locus encoding for INK4b, INK4a, and ARF (also known as p15, p16, and p14, respectively), three tumor suppressors whose function was usually lost or attenuated in human cancers [24]. ANRIL has also been reported to inhibit the expression of a widely known tumor suppressor gene, *INK4b* after its interaction with suppressor of zeste 12 homolog (SUZ12) [8]. In the cells with overexpressed ANRIL, the mRNA and protein levels of INK4b, INK4a, and ARF have been reported to exhibit very low levels, while the anti-proliferative activities of pRB and p53 are then triggered by INK4a, INK4b, and ARF, protein levels [7,9]. p53 is regulated by INK4a and in the absence of p19ARF expression in C2C12 cells results in the loss of the INK4a locus based on the results of a genomic PCR analysis in the study [25]. Our study illustrated that overexpressed ATM acts to reverse the inhibition of INK4b, INK4a, ARF, p53, and pRB induced by the overexpression of ANRIL. Studies have shown that E2F1 induces ANRIL in a transcriptional manner, which leads to a depression in the expression of p16INK4 family, providing an alleviating effect for the p53 and pRB signaling pathways [22]. In this regard, we speculated that ANRIL silencing may possibly prevent retinoblastoma progression via the ATM-E2F1 signaling pathway activation.

Taken together, the key findings of our study suggesting that the silencing of ANRIL can result in suppressed invasion and proliferation, while acting to enhance the apoptosis of retinoblastoma cells by up-regulating the ATM-E2F1 signaling pathway, thus providing a fresh basis for which the treatment of retinoblastoma may be premised upon. Since the localization of lncRNA is beneficial in providing further understanding of its function, the localization of ANRIL on ATM needs further analyzation in future studies. In addition, the underlying molecular mechanism of ANRIL and ATM should be further investigated based on the findings of the present study. Moreover, further experiments should be conducted in order to identify novel therapeutic drugs and provide a new and improved therapeutic strategy for tumor intervention.

## Abbreviations

ANRIL: antisense non-coding RNA in the INK4 locus
ARF: alternate reading frame
CCK-8: cell counting kit-8
EMEM: Eagle’s minimum essential medium
GAPDH: glyceraldehyde-3-phosphate-dehydrogenase
lncRNA: long non-coding RNA
MIC: middle-income country
NC: negative control
OD: optical density
PBST: PBS containing 0.1% Tween-20
PI: propidium iodide
pRB: p53 and retinoblastoma protein
RT-qPCR: reverse transcription quantitative PCR
